# Predictive value of vascular endothelial growth factor polymorphisms on the clinical outcome of renal cell carcinoma patients

**DOI:** 10.3892/ol.2014.2798

**Published:** 2014-12-12

**Authors:** NAN MA, LI-WEI LI, JING-LIANG CHENG

**Affiliations:** 1 Department of Interventional Radiography, The First Affiliated Hospital, Zhengzhou University, Zhengzhou, Henan 4500052, P.R. China; 2 Department of Anesthesia, The First Affiliated Hospital, Zhengzhou University, Zhengzhou, Henan 4500052, P.R. China; 3 Department of MRI, The First Affiliated Hospital, Zhengzhou University, Zhengzhou, Henan 4500052, P.R. China

**Keywords:** renal cell carcinomas, vascular endothelial growth factor, clinical outcome, polymorphism

## Abstract

A cohort study was conducted to investigate the association between vascular endothelial growth factor (VEGF) polymorphisms −2578C/A, −1154G/A and −634C/G and the clinical outcome of renal cell carcinoma (RCC), as well as the interaction of VEGF polymorphisms with tumor stage, metastasis and size. A total of 310 RCC patients were recruited from the First Affiliated Hospital of Zhengzhou University (Zhengzhou, China) between January 2006 and December 2007, and were followed up until December 2012. The association between the three single nucleotide polymorphisms and the overall survival of RCC patients was estimated using Cox’s proportional hazard regression model. The median follow-up duration was 34.7 months and 74 of the RCC patients succumbed due to cancer during the follow-up period. The frequency of the VEGF −2578 AA genotype was significantly higher in patients classed as tumor stages III–IV (odds ratio [OR], 0.47; 95% confidence interval [CI], 0.24–0.95) and larger tumors (longest diameter, >4 cm; OR, 0.44; 95% CI, 0.22–0.89). Furthermore, the frequency of VEGF −634 GG was significantly higher in patients with larger tumors (longest diameter, >4 cm; OR, 0.68; 95% CI, 0.48–0.97). The VEGF −2578 AA genotype was correlated with a 2.96-fold increase in the risk of RCC-associated mortality and was associated with a five-year survival rate of ~25%. Therefore, the present study identified that the VEGF −2578C/A polymorphism may be associated with the prognosis of RCC patients, and may interact with the tumor stage and size.

## Introduction

Renal cell carcinoma (RCC) is a prominent disease, with ~57,760 new cases and ~12,980 mortalities reported worldwide in 2009 (1). Although the majority of patients exhibiting early-stage RCC can be treated surgically, recurrence with distant metastases was observed upon diagnosis in ~25–50% of RCC patients and the five-year survival rate was <20% (2,3). Patients that were diagnosed with the same stage of renal cancer and that received similar treatment to early-stage RCC patients demonstrated a different prognosis, indicating that hereditary factors may contribute to the prognosis of RCC (4,5). Furthermore, previous studies have reported that vascular endothelial growth factors (VEGFs), and platelet-derived growth factors and their receptors may have a role in promoting the pathogenesis of RCC (6,7).

The VEGF gene is a potent endothelial cell mitogen, which consists of eight exons (8). It has been hypothesized that 30 types of single nucleotide polymorphism (SNP) exist in the VEGF gene (8). Three common SNPs, VEGF −2578C/A, −1154G/A and −634C/G, have been widely investigated and identified to be associated with VEGF protein production (9). Furthermore, VEGF −2578C/A, −1154G/A and −634C/G have been associated with the risk or the prognosis of various diseases, such as breast cancer, pancreatic adenocarcinoma, oral cancer and Alzheimer’s disease (10–13).

A previous study indicated that VEGF is overexpressed in RCC tissue when compared with healthy renal tissue (14). Furthermore, therapeutic targeting of VEGF has demonstrated clinical efficacy in the treatment of RCC (15,16); thus, VEGF polymorphisms may be associated with disease progression and prognosis in RCC patients. However, three studies reported inconsistent results regarding the association between VEGF polymorphisms and progression or prognosis of RCC (17–19). Therefore, the current report presents a cohort study investigating the association between VEGF polymorphisms −2578C/A, −1154G/A and −634C/G, and the clinical outcome of RCC patients, as well as the interaction of the VEGF polymorphisms with tumor stage, metastasis and size.

## Patients and methods

### Patients

Patients that were diagnosed with RCC between January 2006 and November 2007 were enrolled in the present study from the First Affiliated Hospital of Zhengzhou University. Patients with a history of pregnancy, malignancy, chemotherapy or radiotherapy were excluded from the present study. All of the biopsy samples were obtained via radical or partial nephrectomy. The RCC tumor stage was determined according to the American Joint Committee on Cancer tumor-node-metastasis staging system (20). The patients in the study were followed up until November 2012, however, six patients were lost to follow-up. Baseline characteristics of all of the patients were obtained using a self-designed questionnaire and medical records. Written informed consent was obtained from all patients and this study was approved by the ethics committee of The First Affiliated Hospital of Zhengzhou University (Zhengzhou, China).

### Polymerase chain reaction (PCR)

All of the patients provided a 5-ml peripheral venous blood sample after consenting to participate in the study. Genomic DNA was extracted using a TIANamp Blood DNA kit (Tiangen Biotech Co., Ltd., Beijing, China) and DNA dissolved in water, according to the manufacturer’s instructions. The presence of VEGF −2578C/A, −1154G/A and −634C/G was determined using PCR combined with a restriction fragment length polymorphism assay (Applied Biosystems, Foster City, CA, USA). The primers and probes for VEGF −2578C/A, −1154G/A and −634C/G were designed using Assay Design 3.1 software (Sequenom Inc., San Diego, CA, USA). The PCR reaction was performed in a 25-μl reaction solution with 25 mM MgCl_2_, each primer and 2 mM deoxynucleotide triphosphates, 1 mmol/l MgCl_2_, 1.25 units Taq polymerase (Takara Biotechnology Co., Ltd., Dalian, China) and 0.5 μl 5X PCR buffer (Takara Biotechnology Co., Ltd.). The DNA was amplified at 95°C for 5 sec, subjected to 40 cycles at 92°C for 40 sec and elongated at 60°C for 40 sec.

### Statistical analysis

All analyses were conducted using SPSS version 16.0 software (SPSS Inc., Chicago, IL, USA). Continuous variables are expressed as the mean ± standard deviation and categorical variables are expressed as frequencies (percentages). The χ^2^ test was used to compare the genotype frequencies between the patients and the controls. The primary end point was five-year survival, which was calculated as the time period from diagnosis to mortality (from any cause), or the last known date that the patient was alive. Survival differences were compared using the log-rank test and multivariate analysis of survival was conducted using Cox’s proportional hazard regression analysis (with hazard ratios [HR] and 95% confidence intervals [CI]) to identify independent prognostic variables. Survival distributions were estimated using the Kaplan-Meier method and assessed using the log-rank test. Two-tailed P-values of <0.05 were considered to indicate a statistically significant difference.

## Results

### Patient characteristics and outcomes

A total of 336 patients with RCC were invited to participate in the present study; 310 patients consented, resulting in a participation rate of 92.26%. The demographic and clinical characteristics of the patients are presented in Table I. The cohort consisted of 206 males (66.45%) and 104 females (33.55%) with a median age of 61.5 years (range, 27.2–81.4 years) upon initial diagnosis. Of the 310 patients, 91.61% exhibited clear cell RCC, 60.32% exhibited stage I–II cancer, 61.29% had a small tumor (longest diameter, ≤4 cm), and 78.39% presented with lymph node or distant metastases. Patients exhibiting clear cell RCC, stage I–II cancer, a small tumor (longest diameter, ≤4 cm) and no metastasis were associated with a longer OS period.

### VEGF genotypes and tumor characteristics

The genotype distributions of VEGF −2578C/A, −1154G/A and −634C/G demonstrated Hardy-Weinberg equilibrium. Conditional regression analysis identified that the VEGF −2578 AA genotype was significantly more frequent in stage III–IV patients (odds ratio [OR], 0.47; 95% CI, 0.24–0.95) and patients with larger tumors (longest diameter, >4 cm; OR=0.44; 95% CI, 0.22–0.89) when compared with the −2578 CC genotype (Table II). Furthermore, the VEGF −634 GG genotype was significantly more frequent in patients with a large tumor (longest diameter, >4 cm) when compared with the −634 CC genotype (OR, 0.68; 95% CI, 0.48–0.97).

### Multivariate analysis

The association between the VEGF genotype and survival with RCC is demonstrated in Table III. The median duration of the follow-up was 33.8 months (range, 2–69 months). Among the 310 patients, 174 patients succumbed due to cancer during the follow-up period, providing a five-year survival rate of 43.87%. The VEGF −2578 AA genotype was significantly associated with poor OS (adjusted HR, 2.96; 95% CI, 1.40–6.53), and the five-year survival rate of patients exhibiting the AA genotype was 25.0% (Table III). However, the VEGF −1154G/A and −634C/G polymorphisms were not significantly associated with the OS of RCC patients. Examination of Kaplan-Meier curves for the VEGF −2578A/C genotypes indicated that the VEGF −2578A/C polymorphism is associated with the overall survival of RCC patients (Fig. 1).

## Discussion

VEGF is involved in the regulation of angiogenesis and is considered to be a potent stimulatory cytokine in tumor angiogenesis, which appears to be key in influencing tumor metastasis and prognosis (21). Previous studies have indicated that polymorphisms in the VEGF gene are associated with various types of cancer, including breast, prostate and gastric cancer. VEGF gene polymorphisms are correlated with various characteristics of cancer, such as susceptibility, tumor grade and OS of cancer (22–24). Three gene polymorphisms, VEGF −2578C/A, −1154G/A and −634C/G, located at the promoter region of VEGF, are involved in altering the gene transcription and expression of VEGF (25). Few previous studies have investigated the association between VEGF −2578C/A, −1154G/A and −634C/G polymorphisms and the prognosis of RCC patients (17–19), thus, the present study is, to the best of our knowledge, the first to identify that the VEGF −2578C/A polymorphism is associated with the prognosis of RCC patients, as well as demonstrating an interaction with the tumor stage and size.

The present study identified that the VEGF −2578 AA genotype is associated with shorter OS period in RCC patients, indicating that the VEGF −2578 AA genotype increases the expression of VEGF and promotes tumor angiogenesis, thus resulting in a higher tumor stage and decreased OS in RCC patients. Therefore, VEGF gene polymorphisms may be critical in altering VEGF expression and influencing the progression of RCC patients. Furthermore, two previous studies reported results that were consistent with the present study, which demonstrated an association between VEGF gene polymorphisms and the prognosis of various diseases (17,26). Hefler *et al* (27) reported that VEGF −634G/C, −1154G/A, and −2578C/A polymorphisms were associated with increased VEGF expression and a shortened OS period in ovarian cancer patients (26). An additional study identified that the −2578 C allele was correlated with increased VEGF production *in vitro* (25). However, reports of an association between −2578C/A polymorphisms and tumor prognosis are inconsistent (21,28,29). For example, Supic *et al* (30) conducted a study of 114 oral squamous cell carcinoma (OSCC) patients and 126 control subjects, and reported a non-significant association between VEGF −2578C/A polymorphisms and the prognosis of OSCC patients (29). The discrepancies between the above-mentioned studies may be due to differences in genetic variant frequencies between individuals with different ethnicities or carcinoma types.

Notably, the VEGF −634 GG genotype is associated with tumor size, although, no association was identified between the VEGF −634C/G polymorphism and the prognosis of RCC patients. One study indicated that the VEGF-634 GG genotype is associated with high serum VEGF levels and reduced OS periods in advanced gastric cancer patients when compared with the CC genotype (21). An additional study identified that the −634 CC genotype was significantly correlated with larger tumor size and higher histological grade (31).

The present study has two limitations. First, the study was conducted in a single hospital in China; thus, it may not be representative of the general population. However, the allele frequencies demonstrated Hardy-Weinberg equilibrium and were similar to the minor allele frequencies obtained from the The National Center for Biotechnology Information database (www.ncbi.nlm.nih.gov/SNP), which indicates that the population of the present study may be representative of the general population. Second, the number of cases analyzed in the present study was relatively small, which may reduce the statistical power to detect differences between the various VEGF allele groups. Therefore, further studies using a large multicenter cohort are required to investigate the association between VEGF gene polymorphisms and the prognosis of RCC patients.

In conclusion, the present study identified that the VEGF −2578C/A polymorphism may be associated with the prognosis of RCC patients, and may interact with the tumor stage and size. Therefore, the present study may aid with predicting the clinical outcome of RCC patients. Further large cohort studies are required to demonstrate the clinical significance of the VEGF −2578C/A polymorphism.

## Figures and Tables

**Figure 1:** Kaplan-Meier curves of renal cell carcinoma overall survival stratified by various VEGF −2578A/C genotypes. VEGF, vascular endothelial growth factor.

**Table I:** Univariate analysis of the demographic and clinic characteristics of 310 renal cell carcinoma patients (age, 61.5 years; range, 27.2–81.4 years).

Variable	Patients, n (%)	Overall survival period, months
Gender		
Male	206 (66.45)	33.5
Female	104 (33.55)	34.6
Tumor histology		
Non-clear cell	26 (8.39)	32.5
Clear cell	284 (91.61)	35.7
Tumor stage		
I–II	187 (60.32)	38.6
III–IV	123 (39.68)	27.4
Tumor size, cm		
>4	120 (38.71)	28.7
≤4	190 (61.29)	36.4
Metastasis		
No	67 (21.61)	35.5
Yes	243 (78.39)	29.2

Tumor size refers to the longest diameter of the tumor. Tumor stage was determined according to the American Joint Committee on Cancer tumor-node-metastasis staging system (20).

**Table II:** Association of VEGF polymorphism with tumor stage, size and metastasis.

VEGF polymorphism	Cases, n	Tumor stage, n		OR (95% CI)^a^	P-value	Metastasis, n		OR (95% CI)^a^	P-value	Tumor size, n		OR (95% CI)^a^	P-value
		
		I–II	III–IV			No	Yes			≤4 cm	>4 cm		
−2578C/A													
CC	145	96	49	1.0 (−)		36	109	1.0 (−)		98	47	1.0 (−)	
CA	113	66	47	0.72 (0.42–1.23)	0.20	23	90	0.77 (0.41–1.45)	0.40	67	46	0.70 (0.41–1.20)	0.17
AA	52	25	27	0.47 (0.24–0.95)	0.02	8	44	0.55 (0.21–1.33)	0.16	25	27	0.44 (0.22–0.89)	0.01
C allele	403	258	145	1.0 (−)		95	308	1.0 (−)		263	140	1.0 (−)	
A allele	217	116	101	0.63 (0.45–0.90)	0.01	39	178	0.71 (0.45–1.08)	0.10	117	100	0.61 (0.43–0.87)	0.00
−1154G/A													
GG	191	117	74	1.0 (−)		44	147	1.0 (−)		120	71	1.0 (−)	
GA	97	57	40	0.90 (0.53–1.53)	0.68	20	77	0.87 (0.45–1.63)	0.64	58	39	0.88 (0.52–1.50)	0.62
AA	22	13	9	0.91 (0.34–2.55)	0.84	3	19	0.53 (0.10–1.92)	0.31	12	10	0.71 (0.27–1.94)	0.45
G allele	479	301	178	1.0 (−)		108	371	1.0 (Ref.)		298	181	1.0 (−)	
A allele	141	73	68	0.63 (0.43–0.94)	0.02	26	115	0.78 (0.46–1.27)	0.30	82	59	0.84 (0.57–1.26)	0.38
−634C/G													
CC	147	91	54	1.0 (−)		34	113	1.0 (−)		98	49	1.0 (−)	
CG	109	63	46	0.81 (0.47–1.39)	0.42	24	85	0.94 (0.49–1.77)	0.83	64	45	0.71 (0.41–1.23)	0.19
GG	54	34	20	1.0 (0.51–2.05)	0.98	9	45	0.66 (0.26–1.56)	0.32	28	26	0.54 (0.27–1.07)	0.06
C allele	403	245	158	1.0 (−)		92	311	1.0 (−)		260	143	1.0 (−)	
G allele	217	131	86	1.01 (0.76–1.33)	0.96	42	175	0.81 (0.52–1.24)	0.32	120	97	0.68 (0.48–0.97)	0.02

a Adjusted for gender and age. Tumor size refers to the longest diameter of the tumor. P<0.05 was considered to indicate a statistically significant difference.

VEGF, vascular endothelial growth factor; n, number of patients; OR, odds ratio; CI, confidence interval; −, no value.

**Table III:** Cox’s proportional hazard regression analysis of VEGF polymorphisms on the survival of renal cell carcinoma patients.

VEGF polymorphism	Cases, n	Mortalities, n	Five-year survival rate, %	Hazard ratio (95% CI)^a^	P-value
−2578C/A					
CC	145	73	49.7	1.0 (−)	
CA	113	62	45.1	1.20 (0.71–2.02)	0.47
AA	52	39	25.0	2.96 (1.40–6.53)	0.00
C allele	403	208	48.5	1.0 (−)	
A allele	217	140	35.3	1.73 (1.21–2.46)	0.00
−1154G/A					
GG	191	104	45.5	1.0 (−)	
GA	97	55	43.3	1.10 (0.65–1.85)	0.72
AA	22	15	31.8	1.79 (0.65–5.43)	0.22
G allele	479	263	45.1	1.0 (−)	
A allele	141	85	39.7	1.25 (0.84–1.87)	0.12
−634C/G					
CC	147	76	48.3	1.0 (−)	
CG	109	63	42.2	1.28 (0.75–2.18)	0.45
GG	54	35	35.2	1.72 (0.86–3.49)	0.10
C allele	403	219	46.7	1.0 (−)	
G allele	217	129	38.7	1.38 (0.98–1.97)	0.06

a Adjusted for gender, age, tumor histology, tumor stage, tumor size and metastasis. P<0.05 was considered to indicate a statistically significant difference.

VEGF, vascular endothelial growth factor; CI, confidence interval; −, no value.
